# Reactive Oxygen Species in Unstimulated Hemocytes of the Pacific Oyster *Crassostrea gigas*: A Mitochondrial Involvement

**DOI:** 10.1371/journal.pone.0046594

**Published:** 2012-10-03

**Authors:** Ludovic Donaghy, Edouard Kraffe, Nelly Le Goïc, Christophe Lambert, Aswani K. Volety, Philippe Soudant

**Affiliations:** 1 Laboratoire des Sciences de l’Environnement Marin, UMR 6539, Institut Universitaire Européen de la Mer, Université de Bretagne Occidentale, Plouzané, France; 2 Department of Marine and Ecological Sciences, College of Arts and Sciences, Florida Gulf Coast University, Fort Myers, Florida, United States of America; Iowa State University, United States of America

## Abstract

The Pacific oyster *Crassostrea gigas* is a sessile bivalve mollusc whose homeostasis relies, at least partially, upon cells circulating in hemolymph and referred to as hemocytes. Oyster’s hemocytes have been reported to produce reactive oxygen species (ROS), even in absence of stimulation. Although ROS production in bivalve molluscs is mostly studied for its defence involvement, ROS may also be involved in cellular and tissue homeostasis. ROS sources have not yet been described in oyster hemocytes. The objective of the present work was to characterize the ROS sources in unstimulated hemocytes. We studied the effects of chemical inhibitors on the ROS production and the mitochondrial membrane potential (Δψ_m_) of hemocytes. First, this work confirmed the specificity of JC-10 probe to measure Δψ_m_ in oyster hemocytes, without being affected by ΔpH, as reported in mammalian cells. Second, results show that ROS production in unstimulated hemocytes does not originate from cytoplasmic NADPH-oxidase, nitric oxide synthase or myeloperoxidase, but from mitochondria. In contrast to mammalian cells, incubation of hemocytes with rotenone (complex I inhibitor) had no effect on ROS production. Incubation with antimycin A (complex III inhibitor) resulted in a dose-dependent ROS production decrease while an over-production is usually reported in vertebrates. In hemocytes of *C. gigas*, the production of ROS seems similarly dependent on both Δψ_m_ and ΔpH. These findings point out differences between mammalian models and bivalve cells, which warrant further investigation about the fine characterization of the electron transfer chain and the respective involvement of mitochondrial complexes in ROS production in hemocytes of bivalve molluscs.

## Introduction

The Pacific oyster *Crassostrea gigas* is a sessile bivalve mollusc which inhabits intertidal zones. This invertebrate species is subjected not only to natural environmental variations but also to pathogenic infections and anthropogenic stressors. Due to their sessile nature, oysters face changing environment while maintaining their homeostasis to survive. Homeostasis in *C. gigas* relies, at least partially, upon cells circulating in hemolymph and infiltrating in tissues, referred to as hemocytes [1]–[3]. Hemocytes are involved in various and numerous physiological functions including nutrient digestion, transportation and distribution [4], [5], as well as shell and tissue repair [6], [7]. Hemocytes also mediate cellular internal defence through accumulation and detoxification of toxicants [8]–[10], phagocytosis and encapsulation of invading, foreign, biological material [11]–[14].

Reactive oxygen species (ROS) are small molecules considered, at least in vertebrates, as involved in internal defence through the elimination of internalized non-self particles such as pathogens [15]–[17]. ROS can, however, interact with host cells’ proteins, lipids, carbohydrates and nucleic acids, irreversibly altering the spatial conformation and function of the impacted molecule [15], [18]. Consequently, the concept of ROS as agents of cellular damage has been widely accepted for a long time.

The production of ROS was previously reported in hemocytes of various bivalve species, including oysters [19]–[24], mussels [25], [26], scallops [27], [28] and clams [29], [30]. Due to the involvement of hemocytes in host defence, ROS production was mostly investigated in the immunological context (Reviewed in [2]). The production of ROS in chemically or biologically stimulated hemocytes was then suggested as NADPH-oxidase related [30]–[33]. In 2003, Lambert et al. [21] first developed flow cytometric methods to investigate the ROS production in hemocytes of bivalves and showed that Pacific oyster hemocytes produce ROS in absence of any kind of stimulation. We recently summarized the ROS pathways commonly accepted but not yet characterized in stimulated bivalves’ hemocytes [2] (Fig. 1).

**Figure 1:** Commonly accepted non-mitochondrial pathways involved in the production of major reactive oxygen species in stimulated bivalve molluscs’ hemocytes, outside the cell membrane (left) and inside phagocytic vacuole (right). Molecular targets of inhibitors (grey boxes) are indicated. NO, nitric oxide; ONOO^−^, peroxynitrite; O_2_^−^, superoxide; H_2_O_2_, hydrogen peroxide; HOCl, hypochloride; NOS, nitric oxide synthase; SOD, superoxide dismutase; MPO, myeloperoxidase. Adapted from Donaghy et al., 2009 [2].

Mitochondria are organelles that generate most of the cell's supply of energy during respiration, through the production of Adenosine TriPhosphate (ATP) by the F_0_F_1_-ATP synthase (Fig. 2). During mitochondrial electron transport, a concomitant transfer of protons (H^+^) across the inner mitochondrial membrane out of the mitochondrial matrix creates and maintains an electrochemical transmembrane potential. The H^+^ gradient is then used by F_0_F_1_-ATP synthase for the phosphorylation of Adenosine DiPhosphate (ADP) to ATP. Such H^+^ motive force is a physico-chemical parameter consisting of two components: a voltage gradient, Δψ_m_, the mitochondrial membrane potential, and a pH gradient, ΔpH [34]. Mitochondria were described as the main sources of ROS production in unstimulated vertebrate cells [35], [36] and there is evidence that mitochondrial production of ROS plays a role in the maintenance of cellular and tissue homeostasis, at least in vertebrates. Indeed, mitochondrial ROS can activate cell proliferation as well as immune and inflammatory responses. Mitochondrial ROS were also reported to be involved in the regulation of glycogen storage, ion-channel function, oxygen sensing, regulation of cellular pH, intracellular trafficking and cell adhesion capacities [18], [36].

**Figure 2:** Hypothetical mitochondrial respiratory chain and sites of ROS production in bivalve molluscs. Molecular targets of inhibitors (grey boxes) are indicated.

The objective of the present work was to characterize the intracellular sources (NADPH-oxidase, nitric oxide synthase, myeloperoxidase, mitochondrial electron transport chain) involved in the production of ROS in unstimulated hemocytes from the marine bivalve species *C. gigas,* through the use of chemical inhibitors. In order to investigate whether ROS production in unstimulated hemocytes is dependent on the mitochondrial activity, we also studied the mitochondrial membrane potential (Δψ_m_).

## Materials and Methods

### Animals

Adult Pacific oysters were collected from the Bay of Brest (04°34′ W 48°21′ N; Brittany, France) from October 2009 to April 2010. No specific permits were required for the described field studies. The location is not privately-owned or protected in any way, and Pacific oyster is not endangered or protected species. Animals were maintained in a flow-through seawater system for a maximum of two weeks before experiments.

### Hemolymph Collection

Hemolymph was withdrawn from the adductor muscle of the oysters using a 2 mL plastic syringe fitted with a 21-gauge needle, through a notch extemporaneously made in the anterior part of the shell. Collected hemolymph was held on ice to reduce cell clumping. Each individual hemolymph sample was microscopically examined to eliminate samples with contaminating particles, such as gametes or tissue debris, and then filtered through an 80-µm mesh. Each experiment was performed on three randomly constituted pools with at least 4 individual oysters for each pool. Pooling of hemolymph was necessitated to obtain enough volume of hemolymph to test the effects of all concentrations of inhibitors and controls simultaneously. In addition, this enabled us to minimize high individual variability.

### Modulators of Intracellular ROS Production

Determination of the involvement of different intracellular ROS sources was performed through the use of chemical inhibitors (Table 1; Fig.1 and 2). All chemicals were purchased from Sigma-Aldrich.

**Table 1:** Intracellular activity and molecular targets of selected chemicals.

Chemicals	Activity
**DPI**Diphenyleneiodonium chloride	Inhibitor of flavoprotein oxidoreductases (*e.g.,* NADPH-oxidase, nitric oxide synthase, mitochondrial complexes I and II)
**Apocynin**4′-Hydroxy-3′methoxyacetophenone	Inhibitor of NADPH-oxidase
**L-NIO**L-N5-(1-iminoethyl) ornitine hydrochloride	Inhibitor of Nitric oxide synthase
**ABAH**4′-aminobenzoic acid hydrazide	Inhibitor of Myeloperoxidase
**FCCP**carbonyl cyanide 4-(trifluoromethoxy)phenylhydrazone	Protonophore. H^+^ equilibrate on both sides of the inner mitochondrial membrane. Dissipation of Δψ_m_ and ΔpH. Uncoupler of oxidative phosphorylation
**Valinomycin**	K^+^ ionophore. K^+^ will cross membranes down the electrochemical gradient. Dissipation of Δψ_m_ and not ΔpH
**Nigericin**	H^+^/K^+^ antiport ionophore. H^+^ equilibrate on both sides of membranes but each H^+^ is replaced by a K^+^. Dissipation of ΔpH and not Δψ_m_
**Rotenone**	Inhibitor of mitochondrial complex I
**Antimycin A**	Respiration inhibitor. Blocks the respiratory chain at complex III between cytochrome b and cytochrome c_1_
**SHAM**Salicylhydroxamic acid	Inhibitor of alternative oxidase (AOX)
**Oligomycin**	Inhibits F_0_F_1_-ATP synthase by blocking the proton channel (F_0_)

Working solutions of chemicals were prepared by serial dilutions of stock solutions. Diluents (DMSO and ethanol) were assessed as non-toxic for hemocytes and concentrations were kept constant between each dilution (Table 2). Final concentrations of chemicals are mentioned in Table 2, text and figures. Briefly, diluted hemolymph (1∶4 in filtered sterile seawater) was incubated with chemical inhibitors and specific fluorescent probes for 30 minutes at 18°C in the dark. After incubation, samples were kept on ice until flow cytometric analyses. Cellular parameters were evaluated using flow cytometer FACSCalibur (Becton-Dickinson) equipped with argon laser 488 nm. Collected data were analysed using WinMDI 2.9 software.

**Table 2:** Tested concentrations of chemicals and final concentration of diluents.

Chemicals	Range of testedconcentrations	Diluent	Final concentration of diluent
**DPI**	0.01–10 µM	10% DMSO	0.1% DMSO
**Apocynin**	0.01–50 µM	25% EtOH	0.25% EtOH
**L-NIO**	0.01–50 µM	dH_2_O (distilled water)	NA
**ABAH**	0.01–50 µM	dH_2_O	NA
**FCCP**	0.01–10 µM	100% EtOH	1.0% EtOH
**Valinomycin**	0.01–10 µM	100% DMSO	0.1% DMSO
**Nigericin**	0.01–10 µM	100% EtOH	0.2% EtOH
**Rotenone**	0.01–10 µM	100% DMSO	0.2% DMSO
**Antimycin A**	0.01–10 µM	100% EtOH	0.2% EtOH
**SHAM**	1–1000 µM	100% EtOH	1.0% EtOH
**Oligomycin**	0.01–10 µM	100% EtOH	1.0% EtOH

### Toxicity of Inhibitors: Assessment of Morphology and Mortality of Hemocytes

Toxicity of inhibitors was determined through the evaluation of morphology and mortality of hemocytes using a double staining procedure including SYBR Green I (1/1000 of stock solution) (Invitrogen) and propidium iodide (10 µg mL^−1^) (PI, Sigma), adapted from Delaporte et al. [37]. Hemocytes of *C. gigas* are composed of two sub-populations, hyalinocytes and granulocytes, whose morphology was based upon relative flow-cytometric parameters, Forward Scatter (FSC) and Side Scatter (SSC) [38]. FSC and SSC commonly measure particle size and internal complexity, respectively. SYBR Green I is a DNA-binding probe which spontaneously penetrates both viable and dead cells. Contrastingly, membranes of viable cells do not allow PI to penetrate; whereas, altered membranes are permeable to PI. Dead cells are characterized by loss of membrane integrity and are, therefore, double stained by SYBR Green I and PI.

### Intracellular ROS Production

Determination of ROS production was performed using 2′7′-dichlorofluorescein diacetate (final concentration 10 µM) (DCFH-DA; Molecular Probes, Invitrogen), a membrane permeable, non-fluorescent probe. Inside hemocytes, the -DA radical is first hydrolyzed by esterase enzymes. Intracellular hydrogen peroxide (H_2_O_2_), as well as superoxide ion (O_2_^•−^; [39], [40]), then oxidizes DCFH to the fluorescent DCF molecule. Oxidation of DCFH can also be mediated by nitrite radicals (NO_2_ or N_2_O_3_) [41]. DCF green fluorescence, detected on the FL1 detector (530/30 nm band pass) of the flow cytometer (FACSCalibur, Becton Dickinson), is proportional to the ROS production. Relative ROS production is expressed as percentage of control condition (*i.e*., without inhibitor).

### Mitochondrial Membrane Potential

Estimation of mitochondrial membrane potential (Δψ_m_) was performed using JC-10 (Interchim; final concentration 5 µM), a membrane permeable fluorescent probe. JC-10 enters selectively into mitochondria and exists as two forms, monomeric or aggregate, depending upon Δψ_m_ and not ΔpH [42], [43]. The JC-10 monomer form predominates in mitochondria with low Δψ_m_ and emits in the green wavelength (525–530 nm). The JC-10 aggregate form accumulates in mitochondria with high Δψ_m_ and emits in the orange wavelength (590 nm). JC-10 forms (monomer/aggregate) can change reversibly. Fluorescence intensities of JC-10 monomers and aggregates were quantified, respectively, by FL1 (530/30 nm) and FL2 (585/42 nm) detectors of the flow cytometer. The JC-10 aggregate/monomer ratio is assumed to be proportional to mitochondrial membrane potential intensity [42], [44].

### Statistical Analysis

Although data are presented as percentage of control (*i.e*., without inhibitor) and expressed as mean (n = 3) ± confidence interval (α = 0.05), statistical analyses were performed on untransformed flow cytometry values. Similarity of variances was first assessed using F-test. In all conditions, no significant difference was observed between variances. The significance of differences between means of control *vs*. each treatment was therefore analysed with *T*-tests (*p*<0.05), using Statgraphics Plus 5 software (Manugistics, Inc., Rockville, MD, USA).

## Results

As previously stated, hemocytes of the Pacific oyster, *C. gigas*, are comprised of two sub-populations [38]. Unstimulated hyalinocytes show lower basal levels of ROS and Δψ_m_ than granulocytes. Both sub-populations reacted similarly to tested inhibitors. The following results reflect the responses of the whole hemocyte population.

### Diphenyleneiodonium Chloride (DPI)

No toxic effect could be detected on hemocytes incubated with DPI in the range of concentrations tested. The detected intracellular ROS formation rate of hemocytes was not altered by DPI from 0.01 to 1 µM (Fig. 3). Incubation of hemocytes with concentrations of DPI higher than 5 µM highly decreased the ROS production, reaching 40% of control at 10 µM. The Δψ_m_ of hemocytes displayed no modification from 0.01 to 0.1 µM (Fig. 3). Application of 0.5 µM of DPI however resulted in a statistically significant major decrease of Δψ_m_ (28% of control condition). The Δψ_m_ was abolished with 5 µM of DPI.

**Figure 3:** Effects of DPI on mitochondrial membrane potential (Δψ_m_) and ROS production of *C. gigas* unstimulated hemocytes. Results are expressed as mean (n = 3) percentage of control (*i.e.*, without inhibitor) ± confidence interval (α = 0.05). An asterisk indicates a statistically significant (t-test, *p*<0.05) difference with the control condition.

### Apocynin, L-N5-(1-iminoethyl) Ornithine Hydrochloride (L-NIO), 4′-Aminobenzoic Acid Hydrazide (ABAH)

In the range of concentrations tested, from 0.01 up to 50 µM, apocynin, L-NIO and ABAH displayed no toxicity toward hemocytes. Incubation of hemocytes with apocynin, L-NIO and ABAH resulted in no modification of detected intracellular ROS, whatever the concentration. Apocynin, L-NIO and ABAH induced no modification of Δψ_m_ in hemocytes (data not shown).

### Carbonyl Cyanide 4-(Trifluoromethoxy) Phenylhydrazone (FCCP)

As expected, the Δψ_m_ of hemocytes decreased very quickly with low concentration of FCCP (0.05 µM) until being abolished at 0.5 µM (Fig. 4A). An inhibition of the ROS production occurred from 0.5 to 10 µM of FCCP (Fig. 4A). Concentrations of FCCP higher than 10 µM were toxic for the hemocytes, as determined by SYBR Green/PI double staining. While mortality of hemocytes in controls was 3.3%, mortality reached ∼20% with 25 and 50 µM of FCCP. Furthermore, morphology of hemocytes incubated with 25 and 50 µM of FCCP was also altered: internal complexity (SSC) decreased to 60% of control (data not shown).

**Figure 4:** Effects of FCCP (A), Valinomycin (B) and Nigericin (C) on Δψ_m_ and ROS production of *C. gigas* unstimulated hemocytes. Results are expressed as mean (n = 3) percentage of control (*i.e.*, without inhibitor) ± confidence interval (α = 0.05). An asterisk indicates a statistically significant (t-test, *p*<0.05) difference with the control condition.

### Valinomycin

As expected, the Δψ_m_ of hemocytes incubated with valinomycin at concentrations higher than 0.05 µM was reduced, and abolished at 1 µM (Fig. 4B). In contrast, the rate of intracellular ROS formation in hemocytes remained constant until 1 µM of valinomycin and then slightly decreased at 5 and 10 µM (Fig. 4B).

### Nigericin

The Δψ_m_ of hemocytes incubated with nigericin (0.01 to 0.5 µM) remained stable and similar to the control condition while incubation with 1 µM of nigericin resulted in a small but significant increase of the Δψ_m_, up to 125% of the control condition (Fig. 4C). Higher concentrations of nigericin then induced a decrease of Δψ_m_, up to 55% inhibition. The detected intracellular ROS formation rate in hemocytes decreased with concentrations of nigericin ranging from 0.1 to 1 µM, reaching a maximum of 30% inhibition (Fig. 4C). Incubation of hemocytes with 5 and 10 µM of nigericin resulted in an increase of ROS production rate.

### Rotenone

Rotenone had no toxicity on hemocytes in the range of concentrations tested. Intracellular ROS and Δψ_m_ of hemocytes were not modified by rotenone and remained similar to the control, whatever the concentrations tested (data not shown).

### Antimycin A

The Δψ_m_ significantly decreased until being abolished from concentrations ranging from 0.1 to 1 µM of antimycin A (Fig. 5). The rate of ROS production in hemocytes was inhibited by antimycin A, reaching 50% inhibition at 10 µM (Fig. 5).

**Figure 5:** Effects of Antimycin A on Δψ_m_ and ROS production of *C. gigas* unstimulated hemocytes. Results are expressed as mean (n = 3) percentage of control (*i.e*., without inhibitor) ± confidence interval (α = 0.05). An asterisk indicates a statistically significant (t-test, *p*<0.05) difference with the control condition.

### Salicylhydroxamic Acid (SHAM)

SHAM induced no toxicity toward hemocytes in the range of concentrations used. The Δψ_m_ was not altered when hemocytes were incubated with SHAM, except for the two highest concentrations (500 and 1000 µM), which resulted in a significant major inhibition of Δψ_m_ (20% of control condition) (Fig. 6A). The detected intracellular ROS were not altered in hemocytes incubated with SHAM.

### Oligomycin

The Δψ_m_ of hemocytes incubated with oligomycin was not altered from 0.01 to 0.1 µM, and then decreased up to 20% of control at 10 µM of oligomycin (Fig. 6B). Incubation of hemocytes with oligomycin reduced the intracellular ROS rates to 50% of control from 0.5 to 10 µM of oligomycin (Fig. 6B). As observed with antimycin A, the inhibition of ROS by oligomycin also statistically occurred prior to the inhibition of Δψ_m_.

**Figure 6:** Effects of SHAM (A) and Oligomycin (B) on Δψ_m_ and ROS production of *C. gigas* unstimulated hemocytes. Results are expressed as mean (n = 3) percentage of control (*i.e.*, without inhibitor) ± confidence interval (α = 0.05). An asterisk indicates a statistically significant (t-test, *p*<0.05) difference with the control condition.

## Discussion

The production of ROS was previously observed in unstimulated oysters’ hemocytes [21] but sources were not yet fully characterized. In the present work, the absence of effect of apocynin, L-NIO and ABAH on ROS production rates suggested that the ROS production in unstimulated hemocytes does not originate from NADPH-oxidase, nitric oxide synthase and myeloperoxidase, contrastingly with Lambert et al. [31] results. Using different chemical inhibitors to investigate intracellular sources of ROS in unstimulated hemocytes, Lambert et al. [31] concluded that about 80–85% of the intracellular ROS production originated from NADPH-oxidase complexes, with the remaining 15–20% supposed to originate from mitochondrial activity. The main reason for misinterpretation by Lambert et al. [31] could have been due to the use of DPI as a specific inhibitor of NADPH-oxidase complexes. DPI is a broad inhibitor of flavoprotein oxidoreductases, including NADPH-oxidase [45], but has also been demonstrated to interfere with nitric oxide synthase [46], mitochondrial respiratory chain NADH reductase (complex I) and succinyl dehydrogenase (complex II) [47]–[50]. In vertebrates, the influence of DPI on ROS production has been described as mostly related to the inhibition of mitochondrial complex I rather than complex II [48], resulting in an increased production of mitochondrial superoxide. In the present work, incubation of hemocytes with DPI inhibited ROS production, as previously reported in human unstimulated monocytes/macrophages [51] and peripheral blood mononuclear cells [50]. Interestingly, incubation of oyster hemocytes with rotenone, an inhibitor of mitochondrial complex I, did not alter Δψ_m_ and ROS production rates as observed with DPI. Rotenone was previously demonstrated to efficiently inhibit complex I in oyster hemocytes [52], but does not seem to alter ROS production rates, as reported here. For its part, DPI may have disturbed markedly mitochondrial activity in hemocytes, as shown by the observed major decrease of Δψ_m_. Reasons for differences in ROS production patterns observed with rotenone and DPI between bivalves and mammalian cells still remain unknown and require further investigation.

Antimycin A inhibits the respiratory chain at complex III between cytochrome b and cytochrome c_1_ [53], [54]. As expected, inhibition of electron transport chain by antimycin A inhibited Δψ_m_ [55]–[57]. Incubation of hemocytes with antimycin A also highly inhibited ROS production. Contrastingly, an increase of ROS production has usually been reported with antimycin A in mammalian cells [58], [59]. In these cells, flow of electrons is inhibited by antimycin A, resulting in a backflow of electrons through complex I which leads to an increase of ROS production [60]. Contrastingly with vertebrates, the electron transport chain of invertebrates is branched with additional terminal oxidases such as the alternative oxidase (AOX) [61]. Studies on marine invertebrates demonstrated the presence of the AOX [62], [63] and the genetic basis for an alternative pathway has been documented in *C. gigas* [61], [64]. AOX accepts electrons directly from ubiquinol and reduces O_2_ to H_2_O, thus representing both a branch in the respiratory chain and an additional terminal oxidase (Fig. 2). By preventing the over-reduction of the respiratory chain, AOX could act to limit ROS generation [61], [64]. AOX could then be hypothesised to being involved in limiting ROS generation due to the backflow of electrons through complex I during incubation of hemocytes with antimycin A. Application of SHAM (inhibitor of AOX) to hemocytes simultaneously incubated with antimycin A did not, however, result in an increase of ROS production (data not shown).

The inhibition of AOX by SHAM alone resulted in no modification of ROS production, suggesting that this oxidase is not spontaneously involved in the ROS production in unstimulated hemocytes. The Δψ_m_ was also not altered by SHAM, except with the two highest concentrations tested. As AOX does not participate in the establishment of the electrochemical gradient, the observed inhibition of Δψ_m_ might be due to a non-specific effect of SHAM at high concentrations. Indeed, it has been suggested that SHAM might inhibit the cytochrome c oxidase (complex IV) [63], the terminal oxidase of the respiratory chain. Inhibition of mitochondrial complex IV could be responsible for the collapse of Δψ_m_ without affecting ROS production.

The final complex of the oxidative phosphorylation machinery is the F_0_F_1_-ATP synthase (complex V) which allows protons to return to the matrix, and uses their potential energy to synthesize ATP [35] (Fig. 2). It has been previously reported in isolated mitochondria that inhibition of complex V may induce an increase of ROS production [65], [66]. Electron transfer driven by complexes I to IV slows down, increasing the “dwell time” for electrons on the complexes and the chance to form superoxide radicals [67]. In the present work, inhibition of complex V resulted in a decrease of ROS production, as reported by Karawajew et al. [68] in a human leukemia cell line. In oyster hemocytes, maintenance of the Δψ_m_ during complex V inhibition might rely on the leak of H^+^ through the inner mitochondrial membrane to the matrix [55], [69]. The two highest concentrations of oligomycin resulted in a drastic decrease of Δψ_m_. An identical pattern of response has been reported in human neutrophils for concentrations higher than 1 µM [70], and might be non-specific and related to additional effects of oligomycin on cells. Oligomycin has been reported to induce hyperpolarization of the cell membranes, resulting in cytoplasmic membrane permeability [71]. Variations in cellular content in ions (e.g., Na^+^, K^+^) might alter the osmotic equilibrium between cytoplasm and mitochondria, leading to the observed decrease of Δψ_m_ and ROS production.

The ionophores nigericin, valinomycin and FCCP were used to study the relative involvement of Δψ_m_ and ΔpH in ROS production from mitochondria. Nigericin inhibits ΔpH without affecting Δψ_m_, while valinomycin decreases Δψ_m_. Lastly, FCCP inhibits both Δψ_m_ and ΔpH by increasing proton leak [72], [73]. Our results confirmed the specificity of JC-10 probe to measure Δψ_m_ in unstimulated hemocytes, without being affected by ΔpH, as reported in mammalian cells [42], [43]. Incubation of hemocytes with valinomycin, which inhibits Δψ_m_, resulted in a 30% reduction of ROS production. Similarly, inhibition of ΔpH by nigericin also decreased ROS production by 30%. In oyster hemocytes, Δψ_m_ and ΔpH then play a role in the production of ROS, and it appears that none seems to dominate. In contrast, Lambert and Brand [74] previously demonstrated that the ROS production in isolated mitochondria from skeletal muscle of rats was more dependent on the ΔpH across the mitochondrial inner membrane than on the Δψ_m_. More recently, Selivanov et al. [73] reported that the pH itself, not the gradient, was an essential factor defining ROS production by the respiratory chain of rat brain mitochondria. Marine bivalve molluscs and terrestrial mammalians such as rats have evolved and exist in totally different environments, in terms of osmolytes and oxygen availability. Oysters are intertidal animals daily exposed to the air for hours. During emersion phases, depletion of available oxygen occurs within the shell [75]. Simultaneously, accumulation of CO_2_ causes a decrease in tissue and hemolymph pH [75], [76]. To date, although no data have been provided to support the fact that such tissue pH decrease affects mitochondrial pH, it is obvious that terrestrial mammalians do not naturally experience such pH variations. This may provide first clues about the observed evolutionary divergence regarding the relative importance of Δψ_m_ and ΔpH for the ROS production.

In summary, the present work evaluated the sources of ROS in unstimulated hemocytes of the Pacific oyster, *C. gigas*. Our results show that ROS in unstimulated hemocytes originate from mitochondria and not from NADPH-oxidase, nitric oxide synthase or myeloperoxidase. Contrastingly with mammalian cells, incubation of hemocytes with rotenone (complex I inhibitor) had no effect on ROS production. Incubation with antimycin A (complex III inhibitor) resulted in a dose-dependent ROS production decrease while an over-production is usually reported in vertebrates. The existence of an AOX in the mitochondrial inner membrane of *C. gigas* might limit over-production of ROS when complex III is inhibited. These findings warrant further investigations about the fine characterization of the electron transfer chain and ROS formation in hemocytes mitochondria of bivalve molluscs, compared with vertebrate models.
